# N1303K (c.3909C>G) Mutation and Splicing: Implication of Its c.[744-33GATT(6); 869+11C>T] Complex Allele in *CFTR* Exon 7 Aberrant Splicing

**DOI:** 10.1155/2015/138103

**Published:** 2015-05-17

**Authors:** Raëd Farhat, Géraldine Puissesseau, Ayman El-Seedy, Marie-Claude Pasquet, Catherine Adolphe, Sandra Corbani, André Megarbané, Alain Kitzis, Véronique Ladeveze

**Affiliations:** ^1^University of Poitiers, “Génétique Moléculaire de Maladies Rares”, 86073 Poitiers, France; ^2^University of Alexandria, Department of Genetics, Aflaton Street, El-Shatby, Alexandria 21545, Egypt; ^3^“Centre Hospitalier Universitaire de Poitiers”, 86021 Poitiers, France; ^4^University of Poitiers, 86000 Poitiers, France; ^5^Saint Joseph University, “Unité de Génétique Médicale”, Faculty of Medicine, Beirut 1104 2020, Lebanon

## Abstract

Cystic Fibrosis is the most common recessive autosomal rare disease found in Caucasians. It is caused by mutations on the *Cystic Fibrosis Transmembrane Conductance Regulator* gene (*CFTR*) that encodes a protein located on the apical membrane of epithelial cells. c.3909C>G (p.Asn1303Lys, old nomenclature: N1303K) is one of the most common worldwide mutations. This mutation has been found at high frequencies in the Mediterranean countries with the highest frequency in the Lebanese population. Therefore, on the genetic level, we conducted a complete *CFTR* gene screening on c.3909C>G Lebanese patients. The complex allele c.[744-33GATT(6); 869+11C>T] was always associated with the c.3909C>G mutation in cis in the Lebanese population. *In cellulo* splicing studies, realized by hybrid minigene constructs, revealed no impact of the c.3909C>G mutation on the splicing process, whereas the associated complex allele induces minor exon skipping.

## 1. Introduction

Cystic Fibrosis (CF) is the most common autosomal recessive genetic disease in Caucasians caused by mutations in the* Cystic Fibrosis Transmembrane Conductance Regulator* (*CFTR*) gene. The prevalence of CF varies and depends on the geographical location [1, 2]. The disease is less frequent in the Arab population in the Middle East region than in Europe [3, 4].

In the Lebanese population, the incidence of both common and rare genetic diseases is relatively high compared to neighbour countries [3] due to the existence of several communities and consanguineous marriage. Around 17% of the patients admitted to the Pediatric Service of American University in Beirut during 1961, 1966, and 1971 were found to suffer from a genetically caused or predisposed disorder [5]. Even though the first Arab CF child was detected in Lebanon in 1958 [6], few accurate pieces of data were presented during the following years to study this disease in the Lebanese population. However, the mutational* CFTR* spectrum of the Lebanese population was roughly elucidated in two previous studies [3, 7]. The major characteristic of this spectrum concerns the c.3909C>G mutation. This widespread mutation appears to have the highest worldwide frequency in Lebanon.

Soon after its identification, the c.3909C>G mutation was characterized by its severity on the pancreas and the variability of the pulmonary status [8]. Despite the low effect in the previous studies, almost all c.3909C>G Lebanese CF patients showed severe pancreatic and pulmonary phenotypes [3, 7]. The presence of a complex allele may aggravate its clinical outcome [9, 10] and can explain the variability of the CF phenotype in CF c.3909C>G patients.

Therefore, to explore the presence of a complex allele, we sequenced* CFTR* genes existing in Lebanon, by recruiting Lebanese c.3909C>G heterozygous and homozygous families. We have detected two variations c.744-33GATT(6) in intron 6 and c.869+11C>T in intron 7 always associated in cis with the c.3909C>G mutation. Therefore, we performed* in cellulo* studies using hybrid minigene constructions to determine firstly the impact of the c.3909C>G mutation on splicing and secondly that of its associated complex allele c.[744-33GATT(6); 869+11C>T].

## 2. Material and Methods

### 2.1. DNA Extraction from Blood Samples

The blood samples were collected in EDTA (ethylenediaminetetraacetic acid) from 7 Lebanese families carrying at least on one allele the c.3909C>G mutation. Genomic DNA was extracted from peripheral blood cells using the QIAamp DNA Blood Mini Kit (Qiagen) according to the manufacturer protocol. The DNA samples were quantified using the Nanodrop 2000 (Thermo).

### 2.2. DNA Amplification

Each of the 27 exons of the* CFTR* gene and their flanking introns were amplified by specific primers. The Pre-PCR reaction (25 *μ*L) consisted of 5 *μ*L of DNA, 2.5 *μ*L of 10x buffer, 2 mmol/L of MgCl_2_, 250 *μ*mol/L of each dNTP, 10 pM of specific primers, and 3 U Taq polymerase. Pre-PCR was performed using a 9700 GeneAmp Thermo Cycler (Perkin Elmer) with the following cycling conditions: initial denaturation (94°C, 2 min), followed by 30 cycles (94°C, 30 sec; 58°C, 30 sec; 72°C, 30 sec), and a final extension step (72°C, 5 min). To eliminate the excess of primers, a step with the ExoSAP (Affymetrix) was realized (15 min at 37°C). The enzyme was directly degraded at 80°C during 15 min.

### 2.3. Direct Sequencing of the* CFTR* Gene

To perform the direct sequencing, PCR reactions were realized on the Pre-PCR product. Sequencing is realized on the purified products using the ABI PRISM Big Dye Terminator TM cycle sequencing Reading Reaction Kit (Applied Biosystem). PCR was performed with the 25 cycles: initial denaturation (96°C, 10 sec), primers hybridization (44°C, 30 sec), and an extension step (60°C, 4 min). Then, purifications of the product were realized by filtration on DyeEx colon (Qiagen) according to the manufacturer protocol. Reactions were run on an ABI PRISM 3100 automatic sequencer (Applied Biosystems). The obtained sequences are aligned and compared to the* CFTR* data base sequences (http://www.genet.sickkids.on.ca/cftr).

### 2.4. Construction of Minigene for Splicing Study

The pTB*Nde*I plasmid (generously provided by F. Pagani) is a strong support to examine the impact of intronic or/and exonic variations on aberrant splicing in transfected mammalian cells. The genomic DNA region of interest, containing a putative splicing mutation, is introduced into the minigene* via* a unique restriction site (*Nde*I) located in a fibronectin intron. The construction and validation of the hybrid minigene used in this study has been described elsewhere [11].

To evaluate the impact of the c.3909C>G mutation on splicing, a PCR fragment, encompassing the 90 bp of exon 24 and 100 pb of each surrounding intron, was amplified from human genomic DNA (Figure 1(a)). Another PCR fragment was amplified to study the impact of the c.[744-33GATT(6); 869+11C>T] complex allele. This fragment contains the 126 pb of exon 7 and nearly 300 pb of each flanking intron (Figure 1(a)). PCR amplifications of these fragments were realized by specific primers described in Table 1.

After plasmid digestion with the* Nde*I restriction enzyme, PCR products were inserted with the DNA ligase (Figures 1(b) and 1(c)). Directed mutagenesis using specific primers was performed to obtain the different minigenes (Figure 1(c)) using the gene tailor site-directed mutagenesis kit (Invitrogen) and specific primers (Table 1). All hybrid minigene constructs were sequenced to verify the correct insertion of WT and mutated DNA fragments (Table 1).

### 2.5. Cell Culture and Transient Transfections

HeLa, HT29, and HEK293 cells were grown in DMEM medium with Glutamax-I (Life Technologies) supplemented with 10% foetal bovine serum (Gibco), 100 units/mL penicillin, and 100 *μ*g/mL of streptomycin in a humidified incubator at 37°C in the presence of 5% CO_2_. Cells were transiently transfected by WT and mutant* CFTR* plasmids using Lipofectamine 2000 (Invitrogen) according to the manufacturer's instructions. At least three independent transfections for each cell line were performed for RNA extraction experiments.

### 2.6. RT-PCR Analyses

Total mRNA was extracted from cell lysates using the RNeasy Mini Kit (Qiagen, Germany) and dissolved in 30 *μ*L of sterile water. cDNA synthesis was carried out at 37°C for 1 h after adjustment of the mixture to contain 5 *μ*L of 5x buffer (Gibco-BRL, France; 250 mmol/L of Tris-HCl pH 8.3, 375 mmol/L of KCl, 15 mmol/L of MgCl_2_), 10 mmol/L of dithiothreitol (Gibco-BRL, France), 1 mmol/L of dNTPs (Roche Diagnostics, France), 2.4 *μ*g of random hexamer primers, 10 *μ*L of RNA, 40 U RNAguard (Amersham Biosciences, Orsay, France), and 400 U Moloney murine leukemia virus (MMLV) reverse transcriptase. The reaction medium was made up to 25 *μ*L with sterile water and the reaction was stopped by incubation at 100°C for 2 min. The PCR reaction (25 *μ*L) consisted of 5 *μ*L of cDNA, 2.5 *μ*L of 10x buffer, 2 mmol/L of MgCl_2_, 250 *μ*mol/L of each dNTP, 10 pM of specific primers for the cDNA (Table 1), and 3 U Taq polymerase. PCRs were performed using a 9700 GeneAmp Thermo Cycler (Perkin Elmer) with the following cycling conditions: initial denaturation (94°C, 2 min), followed by 30 cycles (94°C, 30 sec; 58°C, 30 sec; 72°C, 30 sec), and a final extension step (72°C, 5 min). Amplification products were analyzed by 1.5% agarose gel electrophoresis.

For cDNA obtained from cultured cells, each fragment was purified from a nondenaturing 10% polyacrylamide gel and sequenced with specific primers (Table 1).

## 3. Results

### 3.1. *CFTR* Gene Sequencing in c.3909C>G Patients

The sequencing of* CFTR* 27 exons and their surrounding introns, in the 7 families, confirmed the presence of the c.3909C>G mutation and another mutation in trans, previously determined by the CF30 kit (Elucigene). Furthermore, the sequencing revealed the presence of other different polymorphisms and mutations presented in Table 2. The polymorphism GATT of intron 6 had 6 repeats and the polymorphism c.869+11C>T in intron 7 was present in at least one allele in all the studied patients. The sequencing of exon 7 and part of its surrounding introns of the parental DNA indicated that the GATT(6) and c.869+11C>T polymorphisms are always associated in cis with the c.3909C>G mutation in all the studied patients. Moreover, the allele that does not carry the c.3909C>G mutation has the GATT(7) and no c.869+11C>T polymorphism. Therefore, all the Lebanese patients of this study possess the c.[744-33GATT(6); 869+11C>T; 3909C>G] complex allele.

### 3.2. No Impact of the c.3909C>G Mutation on* CFTR* mRNA Normal Splicing

The sequencing revealed no length difference between the WT and c.3909C>G cDNA, meaning that the c.3909C>G mutation has no effect on splicing regarding the* in cellulo* analyses (Figure 2). Results were identical in all of the three independent transfections in the three tested cell lines.

### 3.3. Splicing Study of the Associated Polymorphisms

Following transient transfections of HeLa, HT29, and HEK293 cells, with the WT (c.[744-33GATT(7); 869+11C]) and mutated (c.[744-33GATT(6); 869+11C>T]) plasmids, mRNA was analysed by RT-PCR and directly sequenced using *β*-globin-specific primers (Table 1). A polyacrylamide gel was used for more precise separation of the resulting fragments (Figure 3(a)). Each fragment was isolated and sequenced with specific primers (Table 1) to determine the different mRNA products.

Polyacrylamide gel shows, for each plasmid construction, two fragments: normal splicing with exon 7 (375 bp) and exon 7 skipping (249 bp). The exon 7 skipping is present in both WT and mutated plasmids. The sequencing, of the different fragments obtained after their purification from the gel, confirmed that the first fragment represents the normal splicing with the complete exon 7 and the second fragment represents that of the exon 7 skipping (Figure 3(b)). This last mRNA is in frame and so induces a shorter fragment than WT-CFTR (−126 bp). Surprisingly, in HEK293 cells, another detected transcript is deleted of one nucleotide (data not shown).

## 4. Discussion

Since its initial identification, the c.3909C>G mutation presented an unclear phenotype-genotype correlation. While the first collaborative study has provided conclusive evidences of the c.3909C>G grave consequences on the pancreas, the severity on pulmonary level remained unpredictable in both homozygous and heterozygous states [8]. In fact, 100% (61 patients) of c.3909C>G/c.1521_1523delCTT and c.3909C>G/c.3909C>G have pancreatic insufficiency, while 72% (23/32 patients) of them present sputum colonization of* P. aeruginosa*. In the Lebanese population, also 100% (8/8) of the same category showed pancreatic insufficiency or growth retardation, and 88% (7/8 patients) revealed pulmonary manifestation [3, 7]. The variable severity regarding the lung disease in c.3909C>G homozygous and heterozygous patients has been previously related to ethnic variation [8]. Environmental factors and/or the presence of a complex allele could modulate the initial consequence of the c.3909C>G mutation. This has led us to recruit all the patients where the c.3909C>G mutation has been detected between 2005 and 2011 in the University of Saint-Joseph genetics laboratory. The complete sequencing of* CFTR* 27 exons and their flanking intronic parts, in all the studied patients, revealed the existence of both c.744-33GATT(6) and c.869+11C>T polymorphisms always associated with c.3909C>G mutation (Table 2). Thus, in this study, we have identified in the Lebanese population the c.[744-33GATT(6); 869+11C>T; 3909C>G] complex allele. This complex allele was already detected in different populations [12, 13].

The examined effect on the c.3909C>G mutation denied the predicted aberrant exon 24 splicing (Figure 2). Despite the early identifications of two associated intronic variations, their impacts on splicing have never been assessed yet neither independently nor in association. The GATT polymorphic region, described in 1990 by Horn et al. in CFTR data base (http://www.genet.sickkids.on.ca), is located in the 5′ flanking region of exon 7 and presents 5 to 7 GATT repeats. The GATT(7) is considered WT since it is the most frequent allele [14]. The c.869+11C>T polymorphism, identified in 1991 by Cuppens et al. in CFTR data base, occurs in the 3′ flanking region of exon 7. In our study, we assessed the influence on splicing, using the minigene assay, in HeLa, HT29, and HEK293 cells, since the severity of the splicing defect may be varied among the cultured cell lines using the same pTB*Nde*I hybrid minigene construct [15]. The WT complex allele (c.[744-33GATT(7); 869+11C]) and the mutated one (c.[744-33GATT(6); 869+11C>T]) uncovered a minor alternative exon 7 splicing in both genotypes. Therefore, the c.[744-33GATT(6); 869+11C>T; 3909C>G] complex allele seems to have no notable influence on the CF phenotype and it is extremely low to explain the variable clinical phenotypes in c.3909C>G patients. However,* in vivo* assessment can validate the splicing outcome and provide justification for further experimental examination of patients samples when available [16].

In conclusion, on the gene level, we identified in the Lebanese population the complex allele associating the c.3909C>G mutation with the c.869+11C>T polymorphism. On the mRNA level, no aberrant splicing was detected with the c.3909C>G. However, we reported minor exon 7 skipping in both WT (c.[744-33GATT(7); 869+11C]) and mutated complex allele (c.[744-33GATT(6); 869+11C>T]). This is unlikely to explain the observed variable phenotype in c.3909C>G patients. However, it is important to note that splicing results differ in function of the cells types. In order to detect the impact of the complex allele on splicing* in vivo*, it is essential to have nasal epithelial cell of homozygote patients with this genotype.

## Figures and Tables

**Figure 1:** Identified complex allele in the Lebanese population and constructions of four hybrid minigenes. (a) The identified* CFTR* complex allele combining the 744-33GATT(6) polymorphism (intron 6), c.869+11C>T polymorphism (intron 7), and the c.3909C>G mutation (exon 24). (b) The pTB*Nde*I plasmid used in the hybrid minigene approach. This plasmid contains a reporter gene used to study the mRNA splicing. The reporter gene contains, at the 5′ end, a promoter/enhancer sequence indicated by the arrow. This is followed by *α*-globin (G1, G2, G3, and G4) and fibronectin (F1 and F2) exons separated by intronic sequences. The fibronectin intronic region, located between F1 and F2, contains a unique* Nde*I restriction site. Fragments of interest can be inserted in this site. (c) The four inserts used in this study. The impact of the c.[744-33GATT(6); 869+11C>T] complex allele on splicing was evaluated by the use of insert 1 (c.[744-33GATT(7); 869+11C]) and insert 2 (c.[744-33GATT(6); 869+11C>T]). Inserts 1 and 2 contain a part of intron 6 (335 bp), exon 7 (126 bp), and a part of intron 7 (326 bp). The impact of the c.3909C>G mutation on splicing was assessed using inserts 3 (WT) and 4 (c.3909C>G). Inserts 3 and 4 contain intron 23 (100 bp), exon 24 (96 bp), and intron 24 (100 bp). Inserts 1, 2, and 3 are obtained from patients and were inserted in the pTB*Nde*I plasmid. Plasmid containing insert 4 was obtained by directed mutagenesis realized on the plasmids containing insert 1.

**Figure 2:** Impact of the c.3909C>G mutation on exon 24 splicing. Sequences of the cDNA were obtained from transfected cells with the pTB*Nde*I minigene plasmid carrying (a) WT or (b) c.3909C>G exon 24* CFTR* minigenes. In both plasmids the sequencing reveals the same transcript, excluding an impact of the c.3909C>G mutation on splicing (the presence of intronic parts in WT and mutated results from plasmid construction and has been detected in the three cell lines).

**Figure 3:** Impact of the c.[744-33GATT(6); 869+11C>T] complex allele on splicing patterns. (a) Polyacrylamide gel showing, for each plasmid construction, the different fragments of cDNA using 2,3*α* and Bra2rev primers on the total cDNA. This polyacrylamide gel shows three independent transfections of the c.[744-33GATT(7); 869+11C] (Lines 1, 2, and 3) and c.[744-33GATT(6); 869+11C>T] (Lines 5, 6, and 7). The results were confirmed in three different cell lines. Two fragments are visible: normal splicing with exon 7 (375 pb) and exon 7 skipping (249 pb). Ladder: *ϕ*X174 DNA/*Bsu*RI (*Hae*III) Marker (Fermentas) was used (Lines 4 and 8). (b) Sequencing of the 375 bp fragment revealing a normal splicing and that of the 249 bp fragment revealing an exon 7 skipping.

**Table 1:** Primers used in amplification and sequencing of studied regions.

Use	Hybridization	Primers
(a) Insert preparation containing the WT exon 24	Intron 23/intron 24	5′ACTTGATGGTAAGTACATGG3′
		5′AGGTATGTTAGGGTACTCCA3′

(b) Insert preparation containing c.[744-33GATT(7);869+11C] or c.[744-33GATT(6);869+11C>T]	Intron 6/intron 7	5′CCAGATTGCATGCTTACTA3′
		5′AGTTACCAATCAGCCTTCA3′

(c) Directed mutagenesis to introduce the c.3909C>G mutation on the pTB*Nde*I plasmid containing the WT exon 24 insert	Exon 24	5′TCTGGAACATTTAGAAAAAAGTTGGATCCCT3′
		5′TTTTTTCTAAATGTTCCAGAAAAAATAAATACTTT3′

(d) Verifying the correct introduction of the inserts in pTB*Nde*I and the correct realization of the direct mutagenesis	Intron fibronectin 1/intron fibronectin 2	5′ACTTCAGATATTATGTCTAGG3′
		5′CCCCATGTGAGATATCTAG3′

(e) Sequencing cDNA of cultured cells	Exon globin 3/fibronectin 2	5′CAACTTCAAGCTCCTAAGCCACTGC3′
		5′AGGGTCACCAGGAAGTTGGTTAAATCA3′

**Table 2:** *CFTR* mutations and polymorphisms identified on each allele of c.3909C>G in Lebanese patients. ^*^No DNA was obtained for the patient number 5 parents; thus the association in cis for the TG(m)T(n) was not determined. As the patient is CF the two detected mutations are in trans.

Individual	Allele	Intron 6	Intron 7	Intron 9		Exon 11	Exon 12	Exon 15	Exon 23	Exon 24	Exon 27
1	1	GATT(6)	c.869+11T	TG(10)	T(9)					**c.3909C>G**	
	2	GATT(6)	c.869+11T	TG(10)	T(9)					**c.3909C>G**	

2	1	GATT(6)	c.869+11T	TG(10)	T(9)					**c.3909C>G**	
	2	GATT(7)	c.869+11C	TG(10)	T(7)			c.2562G	**c.3846G>A**		c.4521A

3	1	GATT(6)	c.869+11T	TG(10)	T(9)					**c.3909C>G**	
	2	GATT(6)	c.869+11T	TG(10)	T(9)	**c.1521_1523delCTT**					

4	1	GATT(6)	c.869+11T	TG(10)	T(9)					**c.3909C>G**	
	2	GATT(6)	c.869+11T	TG(10)	T(9)	**c.1521_1523delCTT**					

5	1	GATT(6)	c.869+11T	10/11TG						**c.3909C>G**	
	2	GATT(6)	c.869+11T	9/7T^*^			**c.1647G**				

6	1	GATT(6)	c.869+11T	TG(10)	T(9)					**c.3909C>G**	
	2	GATT(6)	c.869+11T	TG(10)	T(9)	**c.1521_1523delCTT**					

7	1	GATT(6)	c.869+11T	TG(10)	T(9)					**c.3909C>G**	
	2	GATT(7)	c.869+11C	TG(11)	T(7)	c.1408G					
